The article "Analysis of the Demand for Continuing Education of Nurses in the Department of Infectious Diseases and Its Influencing Factors" was retracted in 2023. Reasons: signs of a paper mill; suspected computer-generated content; unreliable results or conclusions; lack of ethics approval or compliance.

# Analysis of the Demand for Continuing Education of Nurses in the Department of Infectious Diseases and Its Influencing Factors

**DOI:** 10.1155/2022/3743588

**Published:** 2022-09-06

**Authors:** Xiaoqun Pang, Meiling Zhang, Huiyan Pang

**Affiliations:** ^1^Department of Infectious Diseases, The Third Affiliated Hospital of Sun Yat-Sen University, Guangdong, Guangzhou 510630, China; ^2^Department of Operating Theater, The Third Affiliated Hospital of Sun Yat-Sen University, Guangdong, Guangzhou 510630, China

## Abstract

Infection department is unique in working hours, environment, content, methods, and skills requirements, and continuing education plays an important role in stabilizing and improving the professional level of nurses in the infection department. Understanding the needs of nurses in the infection department for continuing education and the possible influencing factors of participating in continuing education and providing a management basis for managers in a targeted way can make the role of continuing education fully play. In this study, according to the characteristics of the Department of Infection, a questionnaire was designed to investigate the continuing education needs of nursing staff in the Department of Infection and analyze the influencing factors. The results show that the nursing staff in the infection department had a greater demand for continuing education. Age, professional title, working life, hospital level, and marital status were the risk factors that affected their demand for continuing education.

## 1. Introduction

In this era of continuous development and progress of society and information explosion, people are paying more attention to health. Unconsciously, patients and society have put forward higher requirements for the quality of care. In addition, with the continuous expansion of the hospital scale, the shortage of nursing staff is more obvious. Most hospitals recruit a large number of new nurses every year to meet the needs of improving the quality of nursing and adapting to the development of the hospital. However, almost all of the nursing staff have such shortcomings as lack of clinical knowledge, insufficient level of operation skills, insufficient clinical experience, lack of communication ability, poor psychological quality, and poor quality of care for high-risk patients, which have affected the patients' medical safety to a certain extent [1, 2]. The infectious disease department is a department with a special position. Due to the particularity of the working environment and working objects, the nurses of the infectious disease department have to face a wide variety of infectious diseases with various transmission routes for a long time [3]. At the same time, the patient's condition is prone to recurrence. So the nursing skills, service attitude, and details of the nursing staff are required to be higher [4]. However, now the main force of the hospital nursing team is the newly recruited nursing staff, and it is particularly important to strengthen their own learning and growth. Nursing staff in the infectious disease department need to continuously learn new knowledge, strengthen and improve their own protection, reduce the harm at work, and ensure the health of themselves and their families to a greater extent, which can effectively reduce the infection rate of patients and reduce the occurrence of nursing errors [5–7].

Continuing nursing education is lifelong nursing education, focusing on the learning of new nursing theories, new knowledge, new technologies, and new methods, which has become the best form of lifelong education and lifelong learning for nurses. With the rapid development of science and technology and the continuous updating of nursing models, the connotation of nursing work has also undergone profound changes. It is necessary for in-service nurses to broaden their knowledge through continuous learning and update the nursing knowledge system in time to meet the needs of modern nursing work [8, 9]. Foreign studies have also pointed out that professional and effective continuing education is crucial to providing safe and high-quality care, regardless of age or seniority, only continuous learning can bring high-quality care to patients. Through the investigation, the nurses of the infection department affirmed the importance of continuing education [10]. However, there are differences in the degree of demand for continuing education among nurses of different ages and qualifications. Only by understanding these differences can we provide a management basis for managers in a targeted manner, and then the role of continuing education can be fully played. Therefore, in order to further understand the demand for continuing education of nurses in different infectious disease departments, our department has carried out relevant research, and the results are reported as follows.

## 2. Materials and Methods

### 2.1. General Information of the Respondents

We randomly selected 160 nurses from the infectious diseases department of 6 general hospitals of Grade III A and 4 hospitals of Grade II Grade A as the survey objects. The nurses participating in this survey are all working in the infectious disease department and have obtained the nurse practitioner qualification certificate.

The survey subjects were all female, with an average age of 28.21 ± 6.35 years and average working years in the infectious disease department 6.54 ± 3.02 years; 13 chief nurses, 20 chief nurses, 35 nurses, and 92 nurses; 75 students with a final degree of bachelor degree or above, 68 students from junior colleges, and 17 students from technical secondary schools; Among them, 102 were from third-class hospitals and 58 were second-class hospitals; marital status, 87 were married and 73 were unmarried.

### 2.2. Research Methods

On the basis of the literature review and characteristics of nursing work in the infectious diseases department, the questionnaire was formed after two rounds of expert evaluation [11]. The questionnaire set up 4 items about continuing education needs, a total of 40 items, and each item has 10 items. The four items are basic knowledge of infectious diseases, common occupational injuries, knowledge of infectious diseases, and disinfection and isolation protection of infectious diseases. Each item is a single-choice question. The options are very need, need, general, and no need, respectively, with 3, 2, 1, and 0 points, respectively. The total score is 120 points. The higher the score indicates the higher the demand. A total of 160 questionnaires were distributed and filled out by anonymous method. A total of 160 questionnaires were collected, and the collection rate and effective questionnaire rate were 100%.

### 2.3. Statistical Processing

The EPI INFO 6.0 software was used to establish the database, and all data were entered twice by a special person. SPSS 13.0 software was used to process and statistically analyze the obtained data, and descriptive statistics, univariate regression analysis, and other methods were used to analyze the data. *P* < 0.05 indicated that the difference was statistically significant.

## 3. Results

### 3.1. Score of Nursing Staff's Demand for Continuing Education in the Infection Department

The average total score for continuing education needs of nurses in the infectious disease department was (89.24 ± 21.96) points, of which the basic knowledge direction of the infectious disease department was (15.36 ± 4.58) points, the common occupational injuries (24.87 ± 4.75) points, the knowledge of infectious diseases (12.71 ± 3.20) points, and disinfection and isolation protection of infectious diseases department (36.30 ± 7.68) points.

### 3.2. Continuing Education Needs of Nurses in the Infectious Disease Department

The survey results show that most of the personnel have a high demand for continuing education, and 69.17% of them have a score of 80 or more. The specific score distribution is shown in Table 1.

### 3.3. Univariate Analysis of Demand for Continue Education of Nursing Staff in the Infection Department

The results of the univariate analysis showed that in addition to educational background, age, professional title, working years, professional title, hospital level, marital status, and other factors had statistically significant differences in continuing education needs between groups. The younger the age, the shorter the working years, the lower the professional title, the lower the hospital level, and the greater the demand for unmarried persons (*P* < 0.05), see Table 2 for details.

### 3.4. Multifactor Analysis on Continue Education Demand of Nursing Staff in the Infection Department

The results of multivariate analysis showed that age, professional title, working years, professional title, hospital level, and marital status were the independent influencing factors of the nursing staff's demand for continuing education in the infectious disease department (*P* < 0.05), see Table 3 for details.

## 4. Discussion

The continuous development of nursing requires that the knowledge system of nurses is constantly updated. The knowledge obtained by school education alone is far from meeting the needs of nursing work, and continuing education as an important way to obtain new knowledge and skills for nurses in service plays a vital role in comprehensively improving the level of nurses' knowledge and skills. At the same time, continuing education for nurses is the need for the development of nursing disciplines and the self-realization of nurses, and it is also a part of lifelong education [12]. Serving nurses generally recognize the importance of continuing academic education. In recent years, with the reform of the medical and health system and the change of the hospital personnel system, education has become the primary condition for nurse employment. In-service nurses are generally aware of the importance of improving their academic qualifications and actively participate in continuing academic education. The ways of continuing academic education are flexible and diverse. Although self-study exams, college entrance examinations, correspondence courses, and online education are all types of national higher education exams, the advantages of self-study exams compared with other types of exams are obvious [13, 14]. Its advantages include quick effect, low cost, and little contradiction between engineering and learning. According to a survey, 65.6% of nurses choose self-study exams as a way to improve their academic qualifications for this reason [15].

The results of this study show that The average total score for continuing education needs of nurses in the infectious disease department was (89.24 ± 21.96) points, which indicates that there is a great demand for continuing education among nurses in the infectious disease department, especially in the disinfection and isolation protection of the infectious disease department and the common occupational injuries in the infectious disease department. As a nurse in the infectious disease department, they need to be in daily contact with biological specimens such as blood, body fluids, secretions, and excreta of infectious disease patients and are under the threat of various viruses. Secondly, the implementation of the strict disinfection system in the infectious disease department, and the various chemical preparations used in disinfection also threaten the health of nursing staff; Furthermore, the closed or semiclosed working environment of the infectious disease department makes it easy for nursing staff to feel depressed, and the worry about acquiring infectious diseases intensifies their psychological burden and damages their mental health [16]. Therefore, it is urgent to cultivate a team of nurses in infectious diseases with a solid theoretical foundation and good mental state through continuing education.

The demand for continuing education of nursing staff in the infection department was analyzed. The results showed that age, professional title, working years, professional title, hospital grade, and marital status were all the influencing factors [17]. Newly recruited nursing staff often have their own weaknesses that are difficult to overcome, mainly reflected in the following points: First, the educational level is low, the foundation is poor, and there are obvious deficiencies in professional theory and logical thinking; they do not have the enthusiasm for active learning and mechanically execute the doctor's orders; Second, there are few opportunities for clinical practice before joining the job. When encountering special patients, they lack confidence and dare not take the initiative to undertake the operation. Over time, the technical operation ability is poor and nonstandard; Third, although they have some theoretical knowledge and nearly a year of internship experience, they are still unable to combine the knowledge they have learned with practice when they encounter emergencies; Nurses are not yet mature in their ability to judge changes in the condition. If they encounter a critically ill patient, they may be at a loss, be in a hurry, panic, and be afraid of facing the situation, and their emergency response ability is poor [18]. Fourth, after the newly recruited nurses started to work independently, due to their lack of knowledge and simple thinking, when faced with family members and patients who have problems or complaints, the nurses do not know if they can communicate effectively, which will make the relationship between nurses and patients tense, which is easy to cause. Nursing disputes arise. Coupled with the particularity of the diseases in our department, the difficulty of intravenous infusion in children with hand, foot, and mouth disease, and the weak protection knowledge and awareness of new nurses, junior nurses often feel physically and mentally exhausted.

In order to reduce the occupational risk of nurses in the infectious disease department, we should carry out corresponding continuing education programs for different groups of people. Continuing education should include the following: (1) Increase the self-protection awareness of nursing staff, adopt a mentoring model, and correct wrong nursing behaviors in a timely manner; (2) Continuously strengthen the professional training of nursing staff, and conduct targeted dissemination of professional knowledge of infection protection; (3) Implement a comprehensive nursing protection mechanism to effectively protect the personal safety of nursing staff [9, 10]. In addition, we should establish an assessment mechanism, and those who fail the assessment should be given counseling and training again, so as to ensure the quality of work and their own safety of the nurses in the infectious disease department [19].

In recent years, the continuous emergence of a variety of educational means has brought vitality to the continuing education of nursing, especially the application of various online education methods, breaking the original classroom teaching methods and emphasizing autonomous learning. Online education, as an extended mode of information distance education, effectively solves the requirements of traditional education mode for time and place. At the same time, online education pays more attention to students' autonomy, and it can also mobilize the classroom atmosphere. And online education has a variety of learning courses, with a wider knowledge coverage, which can better meet the on-the-job nurses' willingness to improve themselves through learning and make learning more efficient [20]. The survey found that most nurses can accept online education to complete on-the-job training, and support the application of online learning to on-the-job continuing education training. Online education can be used as a supplement to continuing education for working nurses and has been shown to be an effective alternative to nurse training. Teachers set clear learning and training tasks according to teaching goals, guide students to discover and analyze problems, and stimulate students' interest in learning; a massive network of teaching resources stimulates students' learning motivation so that students form the habit of autonomous learning and active exploration. In the process of knowledge transmission before class and knowledge expansion after class, students need to make learning plans according to the teaching objectives, and in the process of understanding and mastering the learning content [21]. This method can help nurses gradually develop the learning quality of independent thinking and active inquiry so that they can independently and effectively manage time and monitor the learning effect, and promote the improvement of self-monitoring ability. In the classroom learning process, it is necessary to fully understand the difficulties of knowledge, and fully review and review the knowledge that has been learned. By implementing the case teaching method, discussion teaching method, and group collaboration, group members can form a positive and stable team and establish a harmonious cooperative relationship, to improve the learner's team spirit, communication skills, and other nonintellectual factors. Due to its special working environment in the infectious disease department, nursing staff are in a high-risk working state for a long time, which seriously affects the physical and mental health of nursing staff and the quality of nursing work [22].

To sum up, nursing staff in the infection department had a greater demand for continuing education. Age, professional title, working life, professional title, hospital level, and marital status were the risk factors that affected their demand for continuing education. The deficiency of this study lies in the small sample size. In the future, the sample size can be expanded to further study nurses' demand for continuing education and its influencing factors.

## Figures and Tables

**Table 1:** Distribution of scores of continuing education needs of nurses in the infectious disease department.

Score	120∼100	99∼80	79∼60	59∼40	39 and below
*n* (%)	18 (15.00)	65 (54.17)	36 (30.00)	32 (26.67)	9 (7.50)

**Table 2:** Univariate comparison of continuing education needs among different factor groups.

Indexes	Number of cases	Score	*x * ^2^ value	*P* value
Age			19.768	0.000
> 25 year	83	76.21 ± 13.54		
< 25 year	77	103.28 ± 22.25		

Working years			11.052	0.005
≥ 5 years	78	90.90 ± 12.05		
< 5 years	72	99.84 ± 23.65		

Job title			13.214	0.001
Supervisor nurse and above	68	85.02 ± 17.39		
Nurse	92	95.13 ± 23.74		

Education			3.563	0.158
Bachelor's degree and above	75	87.87 ± 18.35		
College or technical secondary school	85	90.45 ± 22.69		

Hospital grade			16.768	0.000
Tertiary hospital	102	82.45 ± 22.08		
Grade II hospital	58	101.18 ± 23.19		

Marital status			8.254	0.012
Married	87	85.69 ± 19.68		
Unmarried	73	93.47 ± 24.09		

**Table 3:** Logistic regression analysis of continuing education demand.

Indexes	B	SE	Wald Chi-square value	*P* value	OR value
Age	1.765	0.712	15.432	0.017	12.078
Working years	0.952	0.386	9.675	0.048	8.513
Job title	1.172	0.432	10.765	0.035	9.875
Hospital grade	1.825	0.760	14.341	0.009	13.412
Marital status	2.449	0.911	16.349	0.000	16.454
Constant item	−3.203	0.658	11.231	0.003	—

## Data Availability

The data can be obtained from the author upon reasonable request.
